The article "Effect of Bodybuilding and Fitness Exercise on Physical Fitness Based on Deep Learning" was retracted in 2023. Reasons: signs of a paper mill; suspected computer-generated content; unreliable results or conclusions; lack of ethics approval or compliance.

# Effect of Bodybuilding and Fitness Exercise on Physical Fitness Based on Deep Learning

**DOI:** 10.1155/2022/3891109

**Published:** 2022-06-21

**Authors:** Manman Sun, Lijun Wang

**Affiliations:** ^1^College of Sports and Leisure, Xi'an Physical Education University, Xi'an, 710000, Shaanxi, China; ^2^College of Physical Education, Shaanxi Normal University, Xi'an, Shaanxi 710000, China

## Abstract

With the rapid development of society and economy, people's living standards are improving day by day, and increasingly attention is paid to physical health, which has set off a fitness upsurge. The purpose of this paper was to analyze the impact of bodybuilding exercise on physical fitness based on deep learning. It provides a reference for fitness enthusiasts to choose scientific and targeted exercise methods, and provides a theoretical basis for the promotion of bodybuilding and fitness. This paper first gives a general introduction to deep learning and adds image segmentation technology to design experiments for bodybuilding and fitness. The experiment was divided into groups A and B, and control group C. In this paper, recurrent neural network and gated recurrent neural network are introduced to compare and analyze the data, and the stability of data processing with different activation functions is compared. The data results show that under the scientific and reasonable arrangement of exercise conditions, bodybuilding and fitness exercises have a corresponding positive effect on the body shape and posture of the subjects. It is more practical to choose a combination of aerobic and anaerobic exercise. In this paper, based on the deep learning algorithm, compared with the recurrent neural network, the gated recurrent neural network is more suitable for processing sequence problems. In the experimental analysis part, this paper compares and analyzes the experimental results of the data under different activation functions, sigmoid function, and tanh function. It is found that the tanh activation function and the gated recurrent neural network are more stable for data processing. The highest AUC value of the traditional recurrent neural network differs by 0.78 from the highest AUC value of the gated recurrent neural network. The data analysis results are in line with the actual situation.

## 1. Introduction

The national physical quality is not only one of the material foundations for considering the progress of a country and society but also an important manifestation of national strength and social development. However, with the development of society, the way of life and entertainment is diversified. On the one hand, it increases people's income and spare time activities, and enriches people's spare time life and spiritual world. However, on the other hand, economic pressures such as buying a house and unhealthy lifestyles such as staying up late all endanger people's health. Therefore, to meet people's pursuit of physical health, fitness and bodybuilding exercises are increasingly favored by people. Since the effectiveness of bodybuilding and fitness for fat loss has been affirmed by many professionals, many people who have requirements for their own body and posture love bodybuilding and fitness a lot. Fitness bloggers have also sprung up, causing a fitness craze, which has also led to some people's lack of awareness of themselves. It blindly followed the trend and did not take scientific and reasonable fitness methods to exercise. It not only fails to achieve the desired results but also may lead to sports injuries. Therefore, it is necessary to study the impact of bodybuilding and fitness on the body. Deep learning is a network model algorithm emerging in the era of big data. It has demonstrated the superiority of deep learning models for data analysis in many fields such as computer and face recognition.

The article "Effect of Bodybuilding and Fitness Exercise on Physical Fitness Based on Deep Learning" was retracted in 2023. Reasons: signs of a paper mill; suspected computer-generated content; unreliable results or conclusions; lack of ethics approval or compliance.

With the popularity of the Internet, various fitness bloggers' fitness methods have appeared in people's field of vision. However, many enthusiasts do not know enough about bodybuilding and fitness itself. They do not have a scientific and reasonable understanding of how to choose and formulate their own exercise goals and exercise methods, and the arrangement of exercise and exercise is also lacking in pertinence. This also leads to the failure to achieve the expected results after exercising and even sports injuries in severe cases. As a branch of machine learning, deep learning has achieved many achievements in data mining, multimedia learning, recommendation and personalization technology, and other related fields. As an algorithmic method for learning the inherent laws and representation levels of sample data, deep learning is more accurate in studying the impact of bodybuilding and fitness on physical fitness. It has certain theoretical significance for the expansion of the research field of deep learning algorithms. The research on the effect of bodybuilding and fitness on physical fitness in actual exercise can provide a theoretical reference for fitness enthusiasts to choose appropriate exercise plans, which has certain practical significance.

The innovation of this paper is (1) how to choose a more targeted exercise method according to one's own situation when making a bodybuilding and fitness exercise plan. (2) This paper introduces the deep learning algorithm into the research on the impact of bodybuilding and fitness exercise on physical fitness. It can find some hidden laws and characteristics in the research object, which is more valuable for the reference of choosing a scientific fitness method. And this paper compares and analyzes the effect of two different neural network models on data analysis. It breaks the traditional mode of the questionnaire analysis method, and the analysis of data is simpler and more intelligent.

The article "Effect of Bodybuilding and Fitness Exercise on Physical Fitness Based on Deep Learning" was retracted in 2023. Reasons: signs of a paper mill; suspected computer-generated content; unreliable results or conclusions; lack of ethics approval or compliance.

## 2. Related Work

Fitness exercise refers to the use of various exercise methods combined with different forms of exercise in accordance with the principles of human life science. It is a sport that ultimately enhances people's physique, quality of life, and longevity. In foreign countries, many researchers have also conducted research on bodybuilding and fitness exercises and gave interpretations. Dobrescu *T* conducted a sociological study in which bodybuilding can even be used as a professional sport, aiming to promote physical function, psychological development, and esthetic awareness of practitioners [1]. Kashuba V found in the study of the effect of fitness exercise on adult women: in the case of using reasonable water fitness methods, exercise can improve the physical function of women. Therefore, fitness exercise can be regarded as an effective tool for adult women's health improvement and weight management [2].

Deep learning is a general term for a class of pattern analysis methods, and it is also one of the machine learning methods. Deep learning has played an effective role in computer, audio, robotics, information retrieval, and other fields. Yu used a convolutional network algorithm for research to identify Moyamoya disease and predict bleeding events. Combining with research data, he believed that the data obtained through deep learning algorithm analysis is more accurate, sensitive, and specific [3]. Gong *M* studied the detection of changes in synthetic aperture radar images through deep learning. He proposed the feasibility and superiority of deep learning algorithms in different research fields [4]. So, W used the linear activation function of the output layer and the global mean variance of the target features to analyze and process various reverberation times through a deep neural network framework [5]. C Sánchez-Sánchez and Izzo studied the application of deep learning to spacecraft navigation and control systems. In the article, he proposed that the analysis results based on deep learning can allow the design of an on-board real-time optimal control system [6]. Jiang et al. compared deep neural network with other traditional methods and believed that deep neural network is more suitable for video semantic modeling [7]. Various research results have shown the superiority of deep learning algorithms. In different research fields, the types of neural networks are used, such as deep convolutional neural networks [5], and the models are also different.

The article "Effect of Bodybuilding and Fitness Exercise on Physical Fitness Based on Deep Learning" was retracted in 2023. Reasons: signs of a paper mill; suspected computer-generated content; unreliable results or conclusions; lack of ethics approval or compliance.

## 3. Brief Description of Deep Learning Model Algorithm

### 3.1. Deep Neural Networks

Deep learning builds a deep neural network by simulating the neuron activity of the human brain [8]. The basic structure of each neuron is shown in Figure 1.

The output of the previous neuron is the input of the neuron in this layer. Each neuron is similar to a function, receiving n parameters and outputting the result through the calculation of the neuron. However, the last layer of neurons is different from the previous layer, and the output of this layer is generally activated or not activated. The formula is as follows:

(1) $$\begin{array}{c} h\left(m\right)=\left\{\begin{array}{c} 1,\;\text{if}h\left(m\right)>t,\\ 0,\;\text{if}h\left(m\right)\leq t. \end{array}\right. \end{array}$$

Among them, *m* = *X*1, X2, .... Xn, h (m) represents the activation function of the neuron. There are also many types of neuron activation functions, among which the more common is the sigmoid function and the tanh function. The sigmoid function is an activation function commonly used in early multilayer perception [9]. However, when dealing with a relatively large-scale neural network, the tanh function is generally used. The sigmoid function is more commonly used in binary classification problems, but because the gradient of the sigmoid function is very small, when the input is extremely large or extremely small, it will affect the gradient, resulting in a large error in the data. Compared with the sigmoid function, the tanh function has less influence on the gradient [10].

The sigmoid function formula is as follows:

(2) hu=11+e−u.

The tanh function formula is as follows:

(3) $$\begin{array}{c} T\left(x\right)=2h\times 2x-1. \end{array}$$

The sigmoid function image and the tanh function image are shown in Figure 2.

Neither of the two functions completely solves the gradient problem. On this basis, the ReLU function and the Elu function appear in the researcher's field of vision. These two functions can effectively solve the gradient problem as stage functions.

The formula of the ReLU function is as follows:

(4) $$\begin{array}{c} F\left(x\right)=Max\left(0,x\right). \end{array}$$

The Elu function formula is as follows:

(5) $$\begin{array}{c} F\left(x\right)=\left\{\begin{array}{cc} \left(e^{x}-1\right)m, & \text{if}x<0,\\ x, & \text{if}x\geq 0. \end{array}\right. \end{array}$$

The ReLU function image and the Elu function image are shown in Figure 3.

The article "Effect of Bodybuilding and Fitness Exercise on Physical Fitness Based on Deep Learning" was retracted in 2023. Reasons: signs of a paper mill; suspected computer-generated content; unreliable results or conclusions; lack of ethics approval or compliance.

The effect of different activation functions is shown in Table 1.

When a large number of neurons are used as hidden layers, plus the last layer of output neurons, a simple neural network is formed.  Figure 4 is a simple neural network structure.

The figure represents the input layer, hidden layer, and output layer from left to right, and each circle represents a node. The input layer inputs the initial value, and the output layer outputs the result. In the deep neural network algorithm, it is necessary to initialize the weights first, then input the data, and then compare the output layer with the marked value to calculate the error. The output error formula is as follows:

(6) $$\begin{array}{c} E=\frac{1}{2}{\left(T-O\right)}^{2}+I^{2}, \end{array}$$

where *T* represents the tag value *O* represents the output and *I* represents the regularization term.

The traditional neural network model calculation formula is as follows:

(7) $$\begin{array}{c} f=h\left(w\times x+a\right), \end{array}$$

where *f* represents the output node at a certain moment, *x* is the input node at this moment, *w* is the weight, and *h* is the activation function of the neuron. Activation function is a general term. It can be seen from the formula that the output information *f* of the traditional neural network model at different times does not affect each other. However, the influence of fitness exercise on physical quality includes time series. At different time nodes, the degree of influence of bodybuilding and fitness exercise on physical fitness is also inconsistent. Moreover, the impact of fitness exercise on the body is multidimensional. Therefore, traditional neural network models are not suitable for data analysis of the impact of fitness exercise on the body.

The limitations of the traditional neural network model are broken by another neural network model, which is the recurrent neural network model. The peculiarity of recurrent neural networks is their recurrent nature, which makes them more efficient in processing sequence data than traditional neural network models. In sequence data, the training data before and after are not independent, and the sequence of the sequence can also reflect the characteristics of the data, and the recurrent neural network model can handle the ordered data well.  Figure 5 is a data diagram of the recurrent neural network model.

As can be seen from Figure 5, when the recurrent neural network performs data analysis, the hidden layer and the layer can also be transmitted to each other. In the traditional neural network model, each node is connected but independent of each other, although the layers are connected to each other. However, the nodes at the same layer cannot transmit data, and the recurrent neural network model solves this problem well. Data can also be transmitted between nodes in each layer. That is to say, in the recurrent neural network model, the output of the hidden layer is not only related to the output of the input layer. It is also related to the output of the hidden layer at the previous moment [11]. The correlation formula between the value of the hidden layer corresponding to the current node and the value of the hidden layer at the previous moment is as follows:

(8) $$\begin{array}{c} f_{t-1}=h\left(w_{t}+uf_{t-1}\right). \end{array}$$

Among them, *h* is the activation function, and *w* is the weight of the input process.

The article "Effect of Bodybuilding and Fitness Exercise on Physical Fitness Based on Deep Learning" was retracted in 2023. Reasons: signs of a paper mill; suspected computer-generated content; unreliable results or conclusions; lack of ethics approval or compliance.

The input function of the hidden layer of the recurrent neural network at a certain time *t* is as follows:

(9) $$\begin{array}{c} m_{t}{}^{h}=\sum_{i=1}^{i}W_{ih}\times u_{t}^{i},+\sum_{\left(h-1\right)=1}^{h}w_{\left(h-1\right)h}\times n_{t-1}^{h-1}. \end{array}$$

The output function at this time *t* is as follows:

(10) $$\begin{array}{c} n_{t}^{h}=f_{h}\left(m_{t}^{h}\right). \end{array}$$

Among them, *u*_*t*_^*i*^ is the input at time t, *n*_*t*−1_^*h*−1^ is the output at time t − 1, and *w*_*ih*_ is the weight between the input layer and the hidden layer. *w*_(*h* − 1)*h*_ is the weight between the hidden layer at the previous moment and the current hidden layer, and *f*_*h*_ is the activation function of the hidden layer.

The input function of the output layer of the recurrent neural network at a certain time *t* is as follows:

(11) $$\begin{array}{c} m_{t}^{x}=\sum_{h-1}^{h}w_{xh}\times n_{t}^{h}. \end{array}$$

The output function at this time *t* is as follows:

(12) $$\begin{array}{c} g_{t}^{x}=f_{x}\left(m_{t}^{x}\right). \end{array}$$

Among them, *w*_*xh*_ is the weight between the hidden layer and the output layer, and *f*_*x*_ is the excitation function of the output layer.

Similarly, in the cyclic neural network, the error also needs to be calculated. The error formula of the output layer of the cyclic neural network at a certain time *t* is as follows:

(13) $$\begin{array}{c} e_{t}^{x}=g_{t}^{x}-\phi_{t}^{x}. \end{array}$$

At this moment *t*, the hidden layer error formula is as follows:

(14) $$\begin{array}{c} e_{t}^{h}=f_{\left(h-1\right)}\left(m_{t}^{h}\right)\left(\sum_{x=1}^{x}e_{t}^{x}\times w_{xh}=\sum_{\left(h-1\right)=1}^{h}e_{t+1}^{h-1}\times w_{\left(h-1\right)h}\right). \end{array}$$

After the error value is calculated, the partial derivative of each parameter is obtained to obtain the rate of change. The hidden gradient function formula at this time *t* is as follows:

(15) $$\begin{array}{c} e_{t}^{k}=\frac{\partial E}{\partial m_{t}^{a}}, \end{array}$$

where *E* is the error function and *ϕ*_*t*_^*x*^ is the label of *u*_*t*_^*i*^ as shown in formula. At the same time, to better solve the gradient problem and make the error function approximation minimum, it is necessary to use the gradient descent method to process the data [12, 13]. It obtains the minimized loss function and model parameter values to approximately minimize the error function. It needs to be solved iteratively step by step. The gradient descent method formula is as follows:

(16) $$\begin{array}{c} \Delta w_{t}=-\lambda e_{t}, \end{array}$$

(17) $$\begin{array}{c} \Delta w_{t}=w_{t+1}-w_{t}, \end{array}$$

where *λ* is the learning rate and *e*_*t*_ is the gradient at time *t*. This is the general formula of the gradient descent method, but when there are too many calculation samples, the training speed will be slowed down [14], so to make up for this deficiency, the Adagrad algorithm appeared. In this algorithm, a minimum value is added. To ensure that the denominator will not be 0, the calculation formula of the algorithm is as follows:

(18) $$\begin{array}{c} \Delta w_{t}=-\frac{\lambda }{\sqrt{\sum_{t=1}^{t-1}e_{t}^{2}}+\delta }e_{t}. \end{array}$$

The formula for the partial derivative function for each gradient weight is as follows:

(19) $$\begin{array}{c} \Delta E\left(W_{ik}\right)=\sum_{t=1}^{t}e_{t}^{k}\times n_{t}^{i}. \end{array}$$

Combining with the gradient descent method to find the update function of the weightthe formula is as follows:

(20) $$\begin{array}{c} w_{\left(ik+1\right)}=w_{ik}-m\times \Delta E\left(w_{ik}\right). \end{array}$$

Since the cyclic neural network needs to expand the entire network structure and show the characteristics of full connection in the whole neural network [15], more detailed algorithms are needed to solve the gradient problem.

The article "Effect of Bodybuilding and Fitness Exercise on Physical Fitness Based on Deep Learning" was retracted in 2023. Reasons: signs of a paper mill; suspected computer-generated content; unreliable results or conclusions; lack of ethics approval or compliance.

### 3.2. Bodybuilding and Fitness

Fitness and bodybuilding can not only promote the normal development of the human body but also have a positive effect on the body, physical function, and mental health [16]. During adolescence, scientific and appropriate exercise can help promote physical development and greatly improve the physique of adolescents. For ordinary adults, a reasonable arrangement of exercise in leisure time can eliminate part of the impact of life stress on the body and can also delay aging. Bodybuilding and fitness also have related items in sports competitions, which require higher physical fitness of individuals. And they need to devote themselves to sports, but most of them are just public fitness models, using spare time for exercise. Bodybuilding and fitness exercise mainly consists of three parts: stretching exercise, aerobic exercise, and muscle load exercise. When carrying out bodybuilding and fitness exercises, they should scientifically and reasonably arrange the exercises of these three parts according to their own conditions. The selection of the exercise sequence can generally be done with reference to Figure 6.

It can be seen from the figure that a complete fitness exercise should first activate the stretching exercise of the body. After the body adapts to the exercise state, the addition of aerobic exercise can increase the heart rate as part of the warm-up activity. When the body is fully prepared for exercise, it performs muscle-loading exercises to achieve the purpose of shaping the body and finally performs stretching to stretch the muscles to relax the tight muscles.

There are many kinds of bodybuilding and fitness methods for the public, such as aerobics, running, swimming, or exercising with weights such as dumbbells. These sports can generally be divided into aerobic and anaerobic. The more common fitness method is the combination of anaerobic and aerobic. Aerobic exercise is the way to provide the energy required for exercise by aerobic metabolism. Common aerobic exercise mainly includes jogging, rope skipping, swimming, Tai Chi, yoga, aerobics, and others, as shown in Figure 7.

The exercise method carried out in the state of anaerobic function metabolism is anaerobic exercise. Most of the anaerobic exercises are high-intensity and instantaneous sports, such as sprinting, push-ups, weightlifting, muscle strength training, and other long-term muscle contraction exercises as shown in Figure 8.

The bodybuilding and fitness activities of the public are mainly to meet the pursuit of modern people's health. According to a report released by the World Health Organization, the global obesity rate is on the rise. Therefore, in addition to adjusting the diet, proper exercise is also essential. China has also formulated corresponding physical health standards. The normal standards of body mass index, body fat percentage, and vital capacity are shown in Table 2.

### 3.3. Application of Image Segmentation Technology in Human Movement

The application of image segmentation technology in human motion is mainly realized by detecting, identifying, tracking, understanding, and describing the human body in a set of image sequences containing people. Since the human body moves during the motion, this paper chooses the method based on video frame difference to construct the background image.

Assuming that the number of frames is represented by v, M is the sum of the number of frames, and the pixel position is (*a*, *b*). Then, the video frame difference that can reflect the brightness change between adjacent frames is calculated as follows:

(21) $$\begin{array}{c} L_{v}\left(a,b\right)=\left\{\begin{array}{c} c,c\geq D,\\ 0,c<D, \end{array}\right.\\ c=\left|V_{v}+Q\left(a,b\right)-V_{v}\left(a,b\right)\right|. \end{array}$$

Among them *D* represents the threshold for controlling noise removal. The midpoint of the longest segment is selected to fill the corresponding position in the video background among the detected static partsand the reconstructed background obtained is as follows:

(22) $$\begin{array}{c} J\left(a,b\right)=V\left(a,b,H\left(a,b\right)\right),\\ H\left(a,b\right)=\frac{H_{q}\left(a,b\right)+H_{z}\left(a,b\right)}{2}, \end{array}$$

where *H*_*q*_(*a*, *b*) and *H*_*z*_(*a*, *b*) represent the start and end points of the longest stationary sectionrespectively.

The article "Effect of Bodybuilding and Fitness Exercise on Physical Fitness Based on Deep Learning" was retracted in 2023. Reasons: signs of a paper mill; suspected computer-generated content; unreliable results or conclusions; lack of ethics approval or compliance.

Then, we use the background difference method to extract the moving human body. The calculation method is the color value of the pixel point of the current frame minus the color value of the pixel point in the background town, which takes a positive number. After the color difference value is obtained, the value is weighted according to different colors, so as to eliminate the interference of the environment, which can be expressed as follows:

(23) ga,b=ω1FabRed+ω2FabGreen+ω3FabBlue.

Among them, *ω* represents the weight value, and *F*_*ab*_ represents the color difference value of different colors.

We set the global threshold Δ*D* on the image, and the binary image is obtained as follows:

(24) $$\begin{array}{c} J\left(a,b\right)=\left\{\begin{array}{c} \text{background},0;g\left(a,b\right)\leq \Delta D,\\ \text{foreground},0;g\left(a,b\right)>\Delta D. \end{array}\right. \end{array}$$

Double thresholds are used to perform binary processing on the image. First, the low threshold is obtained from the average value of the difference image and the absolute difference of the average value, and the high threshold is obtained by multiplying the ratio of the high and low thresholds by the low threshold. Perform mathematical morphological expansion operation on the low-threshold processed binarized image to obtain the result, and then jointly process the high-threshold processed binary image to obtain a complete moving human body.

This paper will use image segmentation technology to capture the motion of the participants in the experimental part and conduct action guidance.

### 3.4. Impact of Bodybuilding and Fitness Exercises on Physical Fitness Based on Deep Learning

The influence of bodybuilding and fitness exercise on physical quality is multifaceted, and the data of body fat rate, body mass index, and lung capacity in physical function are visualized, and the influence of exercise on the body shows the characteristics of stages. Combined with the deep learning algorithm, a layer of connection GRU between the input layer and the output layer is established between the time points before and after the data; in order to shorten the distance between the relevant characteristics, it includes long-distance data, and another layer is added to allocate the attention coefficient. It is used to reinforce the role of data-focused. The basic structure is shown in Figure 9.

The article "Effect of Bodybuilding and Fitness Exercise on Physical Fitness Based on Deep Learning" was retracted in 2023. Reasons: signs of a paper mill; suspected computer-generated content; unreliable results or conclusions; lack of ethics approval or compliance.

At the same time, to reduce the influence of weights and better solve the error problem, different positional states in the neural network structure of the gated recurrent unit have different effects on the current hidden layer nodes. It can be used to alleviate the problem of vanishing or exploding gradients [17, 18]. It occupies less computer memory resources and is more efficient, which is an advantage compared to recurrent unit networks. The gated recurrent unit neural network structure is shown in Figure 10.

It can be seen from the structure diagram that the gated recurrent unit neural network includes several major structures such as update gate, reset gate, and memory unit [19]. When analyzing the impact on physical fitness, the data are reset and updated according to the time, node, and data type. The function formula is as follows:

(25) $$\begin{array}{c} m_{t}=\text{Tanh}\left(a_{x_{t}}+w_{r}bO_{t-1}\right), \end{array}$$

(26) $$\begin{array}{c} h_{t}=w_{u}O_{t-1}+\left(1-w_{u}\right)m_{t}. \end{array}$$

Among them, *h*_*t*_ is the hidden layer state, *w*_*u*_ is the update gate weight, *O*_*t*−1_ is the input of the hidden layer in the past, *m*_*t*_ is the memory unit, *a* is the input variable, and *b* is the hidden layer parameter.

Considering that the sample data will be unbalanced, that is to say, the proportion of positive and negative samples will change with the test time. This paper introduces AUC to analyze the data [20]. The AUC value is the area under the ROC curve (receiver operating characteristic curve), which represents the ratio of negative and positive cases in the divided instance. The larger the AUC value, the better the effect of fitness and bodybuilding on quality.

## 4. Experiments and Analysis of the Impact of Fitness and Bodybuilding on Physical Fitness Based on Deep Learning

### 4.1. Bodybuilding and Fitness Exercise Combination Design

According to the classification of bodybuilding and fitness, this article compares different combinations of bodybuilding and fitness. It analyzes the impact of different exercise methods on the body. The experiment provides aerobic and aerobic and anaerobic exercise methods. It first controls the duration of each exercise to be 1 hour, and a group of aerobic exercises is one hour. The second group of aerobic exercise and anaerobic exercise is half an hour, and the rest interval between the two groups is the same. It can rest for five minutes to half an hour during exercise to adjust breathing. The specific time arrangement is shown in Figure 11.

The article "Effect of Bodybuilding and Fitness Exercise on Physical Fitness Based on Deep Learning" was retracted in 2023. Reasons: signs of a paper mill; suspected computer-generated content; unreliable results or conclusions; lack of ethics approval or compliance.

Because the exercise program is highly targeted, the arrangement of the exercise program is essential to the experimental results. According to the principles of human life science, the set exercise plan is arranged as shown in Table 3.

This study recruited 20 volunteers between the ages of 22 and 40 who were passionate about bodybuilding and fitness. There are 10 males and 10 females. All subjects have no contraindications that affect sports under the evaluation of professionals, and they can all perform bodybuilding and fitness exercises. To improve the reliability of the data, a control group was added to this experiment, with 5 males and females, and all volunteers aged 22 to 40. The control group did not participate in fitness exercises. The exercise plan is selected according to the body fat rate of the group members and the physical ability of the body. Therefore, this experiment was divided into three groups: A, B, and C. Group A implemented exercise program 1, and group B implemented exercise program 2. This experiment was divided into groups according to the health level of the test indicators, body mass index, body fat rate, and lung capacity before the test. Among them, group A is member with high body fat rate, and group B is member with slightly lower body fat rate and normal range. The various test indicators before participating in the test members are shown in Table 4.

The duration of this experiment was 12 weeks, and subjects were tested for experimental indicators every four weeks. During this experiment, the exercising personnel who participated in the experiment did not participate in other physical exercises except for the exercise during the experiment. The diet is based on a normal diet, not overeating. It also guarantees protein intake during the experiment, guided by professionals during the process. The dietary requirements of the control group were the same as those of the experimental group.

### 4.2. Influence of Bodybuilding and Fitness on Physical Fitness

After three months of exercise, the subject index values are shown in Table 5.

Since the amount of data is not very large, sigmoid and tanh activation functions are selected for comparative analysis. According to the data in the table and the test values in the fourth and eighth weeks, the data results are shown in Figure 12.

The article "Effect of Bodybuilding and Fitness Exercise on Physical Fitness Based on Deep Learning" was retracted in 2023. Reasons: signs of a paper mill; suspected computer-generated content; unreliable results or conclusions; lack of ethics approval or compliance.

As can be seen from the figure, the AUC value increases steadily with the increase of the number of iterations. The highest value of the sigmoid function is higher than the highest value of the tanh function. Compared with the sigmoid functionthe tanh function is more robust in the same neural network model.

Under the same activation function tanh, the comparison of data analysis based on recurrent neural network (RNN) and gated recurrent unit neural network (GRU) models is shown in Figure 13.

It can be seen from the figure that, under the same stable activation function, the AUC value of the gated recurrent unit neural network rises faster and more smoothly, thus proving the effectiveness of the gated recurrent unit neural network based on traditional recurrent neural network optimization.

### 4.3. Control Experiments

To better reflect the validity of the data on the impact of bodybuilding and fitness on physical fitness, the data of the control group were also briefly analyzed. In this paper, the relevant data of the control group C are collected. The values of body mass index, body fat percentage, and vital capacity are also used every four weeks. Under different activation functions, the AUC value changes of GRU and the AUC value changes of different neural network models under the tanh activation function are shown in Figure 14.

According to the graph, it can also be concluded that the tanh function and the gated recurrent neural network model are more stable.

## 5. Discussion

This paper mainly studies the data analysis model based on deep learning, and it applies it to the analysis of the impact of bodybuilding and fitness on physical fitness. This paper not only expands the research field of deep learning algorithms but also increases the data channels for influencing factor analysis. When analyzing data using deep learning algorithms, this article first introduces the application of deep neural networks in different fields. And based on the deep neural network, this paper introduces the optimized deep neural network. In this paper, the algorithm is simply optimized according to the advantages and disadvantages of different neural networks. This paper specifically compares and analyzes the traditional recurrent unit neural network and the gated recurrent unit neural network model under deep learning. This paper derives the utility of using gated recurrent unit neural networks for the analysis of such data. To make the experimental analysis more accurate and the error smaller, this paper compares and analyzes different activation functions in the data analysis model. And in the construction of the neural network model, this paper uses the gradient descent method to optimize the model, to ensure that the error value of the data is approximately the smallest.

The article "Effect of Bodybuilding and Fitness Exercise on Physical Fitness Based on Deep Learning" was retracted in 2023. Reasons: signs of a paper mill; suspected computer-generated content; unreliable results or conclusions; lack of ethics approval or compliance.

Due to the limitations of the experiment, in this data analysis, this paper only uses the gradient descent method and does not compare other optimization algorithms. Under different optimization algorithms, the effect of the model is also different. Therefore, in the future experimental analysis, we can try to use different optimization algorithms to update and train the model to make the data analysis more effective. During the experiment, although the subjects have been restrained according to the relevant requirements, it is difficult to control the suddenness of the physical condition, and there may be errors in the relevant data. Since both body mass index and body fat percentage require body weight data, in terms of city experimental data, body weight is not used as a test indicator alone. Considering that some subjects love fitness, but they do not perform high-intensity exercise. And due to the differences in the physical quality of the volunteers, no anaerobic exercise experiment was carried out in this paper, which is the limitation of this experiment.

## 6. Conclusion

Studies have shown that bodybuilding and fitness exercises can effectively improve the body shape of subjects. In the experiment group A, through aerobic exercise, the body mass index and body fat rate were reduced accordingly, and the burning of body fat disappeared. It effectively plays a role in healthy weight loss. In experiment group B, through the combination of aerobic and anaerobic, the muscle content was significantly increased, and the effect of muscle building was achieved. Both groups of experiments showed that under reasonable and scientific exercise, the lung capacity was also slightly improved. However, the combination of aerobic and anaerobic exercise is more effective than pure aerobic exercise. Therefore, in the selection of the combination of exercise and exercise, it can give priority to the combination of aerobic and anaerobic exercise according to its own physical conditions. In the case of a high body mass index, aerobic exercise with a slightly lower intensity is preferred. In terms of shape, people with a normal body mass index, but relevant requirements can arrange more anaerobic exercise. In the experimental analysis stage, compared with the traditional recurrent unit neural network, the gated recurrent unit neural network is more suitable for the analysis of the impact of bodybuilding and fitness on physical fitness, and the related values are more stable. By comparing and analyzing different activation functions, the tanh activation function is more stable in data analysis.

The article "Effect of Bodybuilding and Fitness Exercise on Physical Fitness Based on Deep Learning" was retracted in 2023. Reasons: signs of a paper mill; suspected computer-generated content; unreliable results or conclusions; lack of ethics approval or compliance.

## Figures and Tables

**Figure 1:** Basic structure of neurons.

**Figure 2:** Sigmoid function image (left) and tanh function image (right).

**Figure 3:** ReLU function image (left) and Elu function image (right).

**Figure 4:** Simple neural network architecture.

**Figure 5:** Recurrent neural network model diagram.

**Figure 6:** Bodybuilding and fitness exercise flow chart.

**Figure 7:** Some common forms of aerobic exercise.

**Figure 8:** Some common anaerobic exercise methods.

**Figure 9:** GRU basic structure.

**Figure 10:** Gated recurrent unit neural network.

**Figure 11:** Movement time design.

**Figure 12:** AUC change graph of GRU under different activation functions.

**Figure 13:** AUC changes in different neural network models.

**Figure 14:** Changes in the AUC value of the model in group C.

**Table 1:** Comparison of activation function effects.

Function type	MAPE	MAE	RMSE
Sigmoid	0.0076	2.16	3.03
Tanh	0.0064	1.93	2.56
ReLU	0.0040	1.14	1.2
Elu	0.0062	1.91	2.51

**Table 2:** Brief list of physical health standards.

Index	Male	Female
BMI	18.5∼23.9	18.5∼23.9
Body fat percentage (%)	15∼18	20∼25
Lung capacity (ml)	3500∼4000	2500∼3500

**Table 3:** Exercise program arrangement.

Frequency (week)	Adapt to the object	Main function
1∼5	Intermediate and advanced	Development force
4∼6	Beginner and intermediate	Build muscle and build strength
5∼7	Fat beginner	Reduce fat and increase muscle endurance

**Table 4:** Numerical table of test indicators for subjects before the experiment.

Group	Number	BMI	Body fat percentage	Lung capacity
A	1	24.3	19.1	3500
	2	24.7	20.3	3500
	3	25.1	20.4	3600
	4	26.3	21.2	3600
	5	24.9	20.3	3500
	6	26.1	25.2	3200
	7	24.6	25.0	2600
	8	25.3	25.6	3000
	9	27.2	25.8	3100
	10	25.6	25.3	3200

B	1	18.2	15	3600
	2	19.1	15.9	3800
	3	22.3	16.7	3600
	4	23.1	18.0	3700
	5	18.4	15.1	3900
	6	21.7	20.1	2800
	7	23.9	23.5	3000
	8	23.6	23.7	3100
	9	23.6	24.3	3200
	10	23.9	24.6	3100

**Table 5:** Numerical table of test indicators after subject experiment.

Group	Number	BMI	Body fat percentage	Lung capacity
A	1	23.9	17.6	3600
	2	24.1	19.7	3600
	3	24.2	19.8	3700
	4	25.0	20.7	3600
	5	23.9	18.3	3900
	6	24.6	23.7	3200
	7	23.7	23.5	2800
	8	24.9	24.8	3000
	9	26.1	25.0	3200
	10	24.2	23.1	3300

B	1	18.5	15.2	3600
	2	19.3	15.7	3900
	3	21.9	16.1	3600
	4	22.9	17.9	3800
	5	18.7	15.3	3900
	6	21.0	20.1	2900
	7	22.6	22.8	3200
	8	23.1	23.1	3100
	9	22.9	23.8	3200
	10	23.1	23.6	3200

## Data Availability

The data underlying the results presented in the study are available within the manuscript.
